RETRACTED

# Evaluation of Mechanical Properties of Materials Based on Genetic Algorithm Optimizing BP Neural Network

**DOI:** 10.1155/2021/2115653

**Published:** 2021-07-19

**Authors:** Tianzeng Liu, Guangping Zou

**Affiliations:** College of Aerospace and Civil Engineering, Harbin Engineering University, Harbin 150001, China

## Abstract

In the 21^st^ century, with the increasingly urgent requirements for lightweight in the fields of aviation, aerospace, and electronics, especially automobiles, many properties of magnesium alloy materials, especially the low-density performance characteristics, have been widely valued. In order to better use magnesium metal materials, it is very important to evaluate its mechanical properties. This article is based on 196 sets of mechanical performance experimental results and related data of AZ31 and AZ91 2 magnesium alloys. Based on data analysis and sorting, take deformation temperature, deformation rate, deformation coefficient, solid solution temperature, and solid solution time as input and take ultimate tensile strength (UTS), yield strength (YS), and elongation (ELO) as output. The 5-8-1 three-layer BP neural network forecast model optimized by the genetic algorithm is used for data training. The training results show that the prediction model can accurately predict the tensile strength, yield strength, and elongation. Compared with the general BP neural network prediction model, the BP neural network based on the genetic algorithm has small discreteness and high fitness: the average error of UTS and YS of AZ31 magnesium alloy is reduced to 0.88% and 3.3%, respectively. The most obvious is that the elongation of AZ31 ELO is reduced, and the error is reduced to 8.1%.

## 1. Introduction

From the emergence of human civilization to today in the 21^st^ century, human social civilization is changing with each passing day, and materials science is also constantly developing. For now, it is urgent to integrate new materials, which will help my country not be controlled by others in the Sino-US trade war [1]. A solid foundation and active development of the new materials industry have been written into the outline of the 12^th^ Five-Year Plan. The green industries led by new materials have taken root in industrial parks in various parts of our country [2, 3]. A series of new materials will surely promote the rapid development of my country's modernization. Magnesium alloy is the lightest metal structural material among the preexisting materials. It has a series of advantages such as small specific gravity, high specific strength, and specific rigidity and is known as the “21^st^ century green environmental protection engineering material.” It has achieved a spurt of development in the fields of energy-saving automobiles, electronic communication products, and aerospace.

RETRACTED

Materials are the material basis for human survival and development. However, there are many materials evaluation and use methods [4]. One of the key points and difficulties of fuzzy comprehensive evaluation at present is how to integrate a multi-index problem into a single-index form, to realize comprehensive evaluation in one-dimensional space. The essence is how to determine the weight of these evaluation indicators. The main methods for determining weights proposed in recent years are subjective and objective. Subjective includes Delphi method, pairwise comparison method, analytic hierarchy process, and serial comparison method [5, 6] and objective includes entropy method, maximum variance method, Fuzzy cluster analysis method, and neural network method. At present, in the field of materials disciplines at home and abroad, computer-aided design and prediction of materials are generally used to provide a valuable reference basis for actual production. Among them, the application research of artificial neural networks is gradually becoming active. In recent years, this method has been used to predict the performance of the materials' mechanical properties [7]. Artificial neural network provides a new way. It does not need to specify basic functions in advance, but based on experimental data, after a limited number of iterative calculations, a mathematical model that reflects the internal connection of experimental data is obtained. In theory, artificial neural network technology can handle arbitrarily complex multivariate nonlinear relationships [8].

The artificial neural network was proposed in the 1940s. After many years of development, its theoretical basis has been perfect. So, it is used in all aspects of life. Because of its powerful ability to deal with nonlinear problems, more and more scholars [9, 10] also applied artificial neural networks to the field of material mechanics analysis. Literature [11] used a neural network model to evaluate the strength of concrete materials and compared it with the results of the least squares fitting formula evaluation. It is concluded that the neural network model can be used to evaluate the strength of ultra-high-strength concrete, and the result is better than the least squares method. Literature [12] used BP neural network to simulate the change rate of dynamic elastic modulus of magnesium alloy material after being corroded by the composite salt solution and found that the measured results are consistent with the predicted results and the average error is 2.08%. The neural network model can more accurately predict the relative dynamic elastic modulus change rate of the magnesium alloy after the corrosion of the composite salt solution. Literature [13] used wavelet analysis method combined with BP neural network and autoregressive integral moving average model to train and predict system signals and random signals during magnesium alloy deformation. Through comparison, it is concluded that the model effectively excavates the effective components contained in the monitoring information, and the forecast accuracy is better. Literature [14] used the neural network to predict the crack resistance of materials based on measured data, and the accuracy of model prediction meets the requirements. Literature [15] established a PCA-BP neural network method and used measured data to predict the structural temperature of large-volume metal materials. The results show that the expected output error is 0.65, indicating that the new model is effective. In literature [16], the yield load and the maximum load of the small punch test are correlated with the yield strength and tensile strength of the material respectively, and the corresponding empirical formulas are given. In literature [17], the initial stage of the load displacement curve of the small punch test is analysed, the slope of the initial stage is correlated with the elastic modulus of the material, the empirical formulas between them are obtained, the third stage of load displacement curve of small punch test is analysed, and the true stress-strain curve and tensile strength of the material are obtained. Nowadays, as computer technology becomes advanced, artificial intelligence is developing rapidly. Because of its convenience and efficiency, the artificial neural network can reduce the complicated derivation process, so it is more and more popular in the analysis of material mechanics.

RETRACTED

This paper is based on 196 sets of mechanical performance test results and relevant data of the two magnesium alloys. It is also based on data analysis and sorting, the alloy elements, deformation temperature, deformation rate, deformation coefficient, solution temperature, solution time, and aging temperature, aging time as input, with tensile strength, yield strength, and elongation as output, and a three-layer BP neural network optimized by genetic algorithm (GA-BP). The network-forecasting model is trained with data to obtain a neural network model with higher accuracy. Using this neural network model can directly provide developers with effective mechanical properties data information under the same process conditions, avoid a large number of experiments, and provide a technical basis for magnesium application research. The main advantages mainly include the following: (1) in the GA-BP model, the nonlinear mapping ability of the neural network, the inference and prediction function of the network, and the global optimization feature of genetic algorithm are used to overcome the problem that the BP algorithm is easily limited to a local minimum and (2) in addition, genetic learning algorithm has the characteristics of global optimization and optimizes the initial weights and network structure of BP network to improve the efficiency of network parameter selection.

## 2. Related Theories and Technologies

### 2.1. Overview of Material Mechanical Performance Evaluation Algorithm

In order to study the durability and mechanical properties of materials, it is necessary to study the evaluation algorithms of the mechanical properties of materials. This paper takes magnesium alloy materials as the main research object and evaluates the mechanical properties of magnesium alloys based on genetic algorithm and BP neural network algorithm. It mainly includes magnesium structure analysis, mechanical experiment design, construction of mechanical performance evaluation model, and experimental result analysis.  Figure 1 shows the overall structure of the magnesium alloy material mechanical performance evaluation algorithm.

Magnesium and most magnesium alloys have a hexagonal close-packed structure (hcp). At room temperature, the lattice constant (*c* = 0.5119 nm, *a* = 0.3202 nm, *c*/*a* = 1.623 nm) and the standard hexagonal close-packed structure (*c*/*a* = 1.633) are very close; as the temperature rises, the increase of the slip system and the combined effect of the twinning effect increase its shaping, which is formed by extrusion rolling and forging [18, 19]. The main plastic deformation of magnesium alloy is slip, followed by twinning. For magnesium alloys with a close-packed hexagonal structure, twin deformation is particularly important, and its shear is also along a specific crystal direction; whether twinning occurs is related to the symmetry of the crystal. The slip in the magnesium alloy crystal only occurs in the crystal inclined to the tensile stress direction, so the plastic deformation of the magnesium alloy is often slip and twinning. Because of the interaction, at the same time, the factors affecting the plastic workability of magnesium alloys include deformation temperature, strain rate, stress state, and texture. Commonly used elements of magnesium alloys mainly include Al, Zn, Mn, Si, and impurity elements (Fe, Cu, and Ni). Of course, the distinction between impurity elements and alloying elements is relative, and alloying elements may become harmful elements in some cases. In some cases, harmful elements can become beneficial elements.

RETRACTED

### 2.2. Theoretical Basis of Neural Networks

Neurons are the most basic unit of the human brain that can receive and process information. The brain can continuously adapt to changes in the external environment through self-organization and self-learning. Neuronal cells are the carriers of human learning and memory. Their morphology is very different but their functional structures are similar. The information in biological neurons is transmitted from dendrites to neuron cells in the form of stimulus signals. After the information is processed by the cell body, the axons transmit the signals. When the intensity of the stimulus signal is higher than a certain value, a nerve impulse meridian is generated. When the intensity of the stimulus signal is lower than a certain value, no nerve impulse is generated.

Artificial neural network (ANN) is an arithmetic model established by humans to deal with the function and structure of the brain [20–22]. It has similar functions to the human brain. For example, learning, association, memory, and other functions are important ways to simulate human intelligence. Similar to the way of human memory, a neural network is a model that solidifies a huge number of weight domain values between separated nodes to form the memory of the network. BP neural network is a kind of multilayer feedforward network. It uses the gradient descent method to train the weight range of the neural network through backpropagation and solves complex nonlinear problems in engineering. It is regarded as the starting point of neural network research in the sense of modern engineering [23]. BP neural network is also called error backpropagation neural network or error back learning algorithm. It uses the back feedback of errors to adjust the weight domain value layer by layer to adjust the network itself. At present, the most widely used neural network basically uses the BP network and its variants. Its structure is shown in Figure 2. The standard BP neural network adopts that when the output error is within the set error range, or the number of error steps is greater than the set value, or the set maximum number of learning times or learning time is reached, the learning process is terminated and the network training ends.

For the three-layer BP neural network shown in Figure 2, set the input vector *A*=(*a*_1_, *a*_2_,…, *a*_*n*_); the hidden layer input vector *B*=(*b*_1_, *b*_2_,…, *b*_*p*_), output vector *C*=(*c*_1_, *c*_2_,…, *c*_*k*_); and output layer input vector *L*=(*l*_1_, *l*_2_,…, *l*_*q*_). The output vector *S*=(*s*_1_, *s*_2_,…, *s*_*q*_); the weights of input-implicit-output are *w*_*ij*_ and *w*_*jt*_, respectively; the thresholds of the two implicit output layers are *θ*_*j*_ and *θ*_*t*_, respectively; the expected output vector *Y*=(*y*_1_, *y*_2_,…, *y*_*q*_); the number of samples *k*=1,2,3,…, *m*; and the excitation function adopts an *S*-type function.

RETRACTED

The learning steps of the BP neural network are as follows. Step 1: neural network initialization. In the range of (−1, 1), the connection weight and domain value of the hidden layer of the input layer and the output layer are randomly assigned. Step 2: use a random method to extract the *k-*th input sample data and the corresponding expected output sample data *A*(*k*)=(*a*_1_(*k*), *a*_1_(*k*),…, *a*_*n*_(*k*)), *Y*(*k*)=(*y*_1_(*k*), *y*_1_(*k*),…, *y*_*n*_(*k*)) and provide them to the neural network. Step 3: use the connection weights and thresholds of each layer to calculate the input *b*_*j*_ and output *c*_*j*_ of each neuron in the hidden layer and the input *l*_*t*_ and output *s*_*t*_ of the output layer:

(1) $$\begin{array}{c} b_{j}=\underset{n⟶\infty }{\lim}\overset{n}{\underset{i=1}{\sum }}w_{ij}a_{i}+\theta_{j},\\ c_{j}=g\left(b_{j}\right),\\ l_{t}=\underset{p⟶\infty }{\lim}\overset{p}{\underset{j=1}{\sum }}w_{jt}b_{j}+\gamma_{t},\\ s_{t}=g\left(l_{t}\right). \end{array}$$

Step 4: use the expected output and actual output of the network training to calculate the neuron errors *d*_*t*_^*k*^ and *e*_*j*_^*k*^ of the output layer and the hidden layer with the established empirical formula:

(2) $$\begin{array}{c} d_{t}^{k}=\frac{\left(1+s_{t}\right)}{\left(y_{t}^{k}+s_{t}\right)}\;t=1,2,\ldots ,1,\\ e_{j}^{k}=\underset{q⟶\infty }{\lim}\overset{q}{\underset{t=1}{\sum }}\frac{d_{t}w_{jt}}{\left[\left(1-c_{j}\right)c_{j}\right]}\;j=1,2,\ldots ,p. \end{array}$$

Step 5: use the neuron error *d*_*t*_^*k*^ obtained in each layer of the output layer and the output of each neuron in the hidden layer to correct the connection weight and threshold between the hidden-output layers:

(3) $$\begin{array}{c} w_{jt}\left(N+1\right)=w_{jt}\left(N\right)-\alpha \cdot d_{t}^{k}\cdot c_{j},\\ \theta_{t}\left(N+1\right)=\theta_{t}\left(N\right)-a\cdot d_{t}^{k}\;0<\alpha <1. \end{array}$$

Step 6: use the error *e*_*j*_^*k*^ of each unit of the hidden layer and the input of each neuron of the input layer to correct the connection weight and threshold between the input and the hidden layer:

(4) $$\begin{array}{c} w_{ij}\left(N+1\right)=w_{ij}\left(N\right)-\beta e_{j}^{k}a_{i}^{k},\\ \theta_{j}\left(N+1\right)=\theta_{j}\left(N\right)-\beta e_{j}^{k}\;0<\beta <1. \end{array}$$

Step 7: randomly select from the remaining training samples and provide it to the network for training, and then return to Step 3 until the training of *m* training samples is completed. Calculate the global error *E*:

(5) $$\begin{array}{c} E=\underset{m⟶\infty }{\lim}\frac{1}{2m}\overset{m}{\underset{k=0}{\sum }}\overset{q}{\underset{t=1}{\sum }}{\left[y_{t}\left(k\right)+s_{t}\left(k\right)\right]}^{2}. \end{array}$$

Randomly select a training sample and input it into the neural network that sets the maximum number of calculations and set the error and training time for training. When any one of the conditions is met, the training ends. You can judge whether the established neural network meets the requirements by comparing the number of training times, training time, and errors.

RETRACTED

### 2.3. Overview of Genetic Algorithm

It is generally believed that the genetic algorithm (GA) is one of the three components of an evolutionary algorithm. A method imitates the genetic mechanism of nature and randomizes the global search for the optimal solution. The basic idea is based on Darwin's theory of evolution and Mendel's genetics. Doctrine and the search and optimization process are completed by iteration, which has become an important discovery of human bionics and has a wide range of use value [24]. The excellent self-learning ability of the genetic algorithm is an advantageous tool for solving complex relationships. Because genetic algorithm has no continuity and nondifferentiability for the required problems, it requires reference to the research results of biological genetics. The genetic algorithm aims at the global solution space. The continuous evolution of the solution space realizes the global search and optimization, so the genetic algorithm is very effective and promising in solving complex artificial intelligence problems.

The genetic algorithm is a kind of random search and optimization algorithm established by simulating the genetic and long-term evolution process of the above-mentioned biological population. It consists of three basic operators. Selection, crossover, and mutation are called genetic operations. The individuals in the genetic space are chromosome; the basic component of an individual is a collection of genetic genes. A collection of individuals is called a population. The adaptability of an individual to the environment is expressed by fitness. Large adaptability indicates strong adaptability of the individual because fitness is an individual survival opportunity in the population [25]. Therefore, the form of fitness function directly determines the evolutionary behaviour of the group. The genetic algorithm is an iterative optimization process. The genetic operation encodes sample data to generate a population, then determines the fitness function, and then performs crossover and mutation operations on the generated population. After the continuous operation of the genetic algorithm, new generations of new generations are generated. The genetic algorithm solving process is shown in Figure 3.

RETRACTED

Crossover is the process of gene recombination that imitates sexual reproduction in nature. Two individuals are randomly selected from a population with a higher fitness for random pairing, which is called the parent. According to the selected crossover method and crossover probability, the individual genes are exchanged to form a pair of offspring. Crossover methods include one-point crossover and multipoint crossover. The process of randomly swapping two genes at the same position from the same parent to produce two new offspring is called one-point crossover. The crossover process of 5678 loci on the parent gene chain is shown in Figure 4(a). Assuming that the fitness *f* of an individual is represented by the square of its binary number symbol string converted into a decimal integer, the fitness of the parent before the crossover is 29^2^ = 841 and 146^2^ = 21316 and the fitness of the offspring after the crossover is 18^2^ = 324 and 157^2^ = 24649. It can be seen that the offspring's gene chain is inherited and reorganized by the parent, and the offspring may surpass the parent to reflect evolution. The principle and method of the multipoint crossover are the same as those of one-point crossover. A crossover algorithm is an important feature of the genetic algorithm, which distinguishes it from other algorithms.

Mutation operation is an auxiliary method used to generate new individuals in genetic algorithms. It refers to the process of replacing some genes of other individuals with part of the gene string of any individual in the population to form a new individual. The mutation process is shown in Figure 4(b). It is also possible to mutate a given chromosome bit string *s*_1_=*a*_1_*a*_2_ … *a*_*L*_ by algebraic method, as follows:

(6) $$\begin{array}{c} F\left(p_{m},x\right):\;a_{i}^{\prime }=\left\{\begin{array}{cc} 1+a_{i} & \text{if }x_{i}\leq p_{m}\\ a_{i} & \text{if }x_{i}>p_{m} \end{array}\;i=1,2,\ldots ,L\right). \end{array}$$

New individuals *s*_1_′=*a*_1_′*a*_2_′ … *a*_*L*_′ are generated. Among them, *x*_*i*_ is the uniform random variable corresponding to the gene, *x*_*i*_ ∈ [0,1].

## 3. Evaluation Model of Mechanical Properties of Magnesium Alloy Materials Based on GA-BP Neural Network

### 3.1. Collection, Sorting, and Analysis of Training Data of Mechanics Evaluation Model

The data used in the establishment of AZ31 and AZ91 BP neural network-forecasting models are all derived from experimental data. To select useful data samples from the obtained data, first analyse, sort, and count. Based on ensuring the accuracy and feasibility of the model, the established model is determined to be AZ31 and AZ91 magnesium alloys with sufficient data to be deformed by the extrusion process, and the BP neural network model of the corresponding composition, process, and performance is established. In order to unify the standard as much as possible, the data obtained in the literature under the same conditions are used. After further sorting and classification, 196 groups of AZ31 and AZ91 magnesium alloy data with relatively large correlation have been sorted out. Each group of data here includes a data set of composition, process, heat treatment, and mechanical properties.

RETRACTED

AZ31 and AZ91 are magnesium alloys; the main parameters are extrusion temperature, extrusion rate, and extrusion ratio; the commonly used heat treatment methods mainly include solution treatment; and the main parameters are solution temperature and solution time. After solution treatment, the cooling methods include water-quenching, oil quenching, and air-cooling. Due to the diversity of these data, it is difficult to quantify, so they are unified as the data obtained by the air-cooling used in the experiment of the research group.  Table 1 is the statistical analysis of processing parameters and processes in AZ31 and AZ91 magnesium alloy samples.

In the collected mechanical property data of AZ31 and AZ91 magnesium alloys, they are basically the mechanical property data at room temperature. There is a small amount of high-temperature performance data, but there is no low-temperature performance data. This may be related to the current research status of magnesium alloys. Therefore, the data used in this topic are the mechanical property data at room temperature and the data tested in the experiment. Statistical analysis of the mechanical properties of AZ31 and AZ91 magnesium data samples includes yield strength 196 groups, tensile strength 188 groups, and elongation 161 groups.

### 3.2. Prediction of Mechanical Properties and Establishment of BP Neural Network Model

The general BP neural network is composed of an input layer-hidden layer-output layer. The number of hidden layers determines the accuracy of the neural network and the amount of calculation. However, the three-layer BP neural network can complete most of the actual problems, and any continuous function can be used for convergence calculations. Therefore, a three-layer neural network is used when establishing the AZ31 and AZ91 mechanical models. If the number of hidden neurons is too small, the error of the neural network will be too large, and the significance of model building will be lost. If the number of hidden neurons is too large, the amount of calculation will be too large and the training time will be too long or even unable to converge, thus forming an endless loop. According to the empirical formula, the neural network structure is finally determined to be 5-8-1. The three-layer BP neural network structure is shown in Figure 5. Using the training program formed by the above conditions, the corresponding AZ31 and AZ91 magnesium alloy ultimate tensile strength (UTS), yield strength (YS), and elongation (ELO) BP neural network models were established respectively.

RETRACTED

### 3.3. Model Optimization Based on Genetic Algorithm

The BP neural network itself has its own shortcomings, mainly for the training uncertainty of complex problems in the training process, which is specifically manifested in the following two aspects. On the one hand, it cannot be trained. In the BP neural network training process, if the default parameters given by MATLAB are too large, it may cause some weighted average values to be too large, which makes the activation function deviate from its working area, which makes the function's weight adjustment invalid for the network. In order to avoid this phenomenon, firstly choose a smaller initial weight and secondly use a smaller one. Learning rate: this choice will increase training time. On the other hand, it is easy to choose a local minimum. BP neural network uses the gradient descent method to make the network weights converge to a solution. However, the global minimum solution of the hyperplane cannot be obtained. The reason is that the training gradually reaches the minimum error of the error slope from a certain starting point. However, for a complex BP neural network, its error function is a curved surface in a multidimensional space. Training may get a minimum value, and this minimum value only represents a region and cannot represent the global minimum. The genetic algorithm uses a parallel global search method. The artificial neural network has the characteristics of self-learning. Using a genetic algorithm to optimize the BP neural network model can make the newly established learning algorithm have the advantages of both.

In the process of optimizing the BP neural network using a genetic algorithm, the genetic algorithm performs circular selection, crossover, mutation, and fitness calculation operations on the sample data. Through simulation experiments, it is determined that the optimal fitness of the population reaches the maximum target fitness value during the 80 generations of evolution. Obtain the optimal weights and thresholds, and use the optimal initial weights and thresholds to construct a BP neural network to train the network.

RETRACTED

According to the flowchart of BP neural network optimization by the genetic algorithm shown in Figure 6, the optimization process of genetic algorithm for BP neural network includes the following aspects: (1) adjust the number of neurons in the hidden layer of the neural network according to the size of the error between the actual output and the expected output. (2) Encode the data to generate the initial population, discretize to form chromosomes, perform cross-mutation on the data, and determine the optimal weight threshold. (3) Determine the fitness function. The fitness function represents the environmental adaptability of each individual in the population. This paper uses the error square sum EEEE of the BP neural network training sample as the fitness function; that is, the genetic algorithm should be carried out in the direction of increasing fitness. (4) Genetic algorithm function extreme value optimization is mainly divided into two steps: BP neural network training, fitting, and genetic algorithm extreme value optimization.

## 4. Experimental Results and Analysis

### 4.1. Mechanical Properties of Materials Evaluation Model Validation Results Analysis

First, the performance of the built model of material mechanics evaluation is verified, and the common evaluation function is used to verify the performance of the established BP neural network and the BP neural network optimized by the genetic algorithm. The experimental results are shown in Figure 7.

It can be seen from Figure 7(a) that after the estimation of the GA-BP neural network, although there will be many minima areas, the population will eventually call out the minima to find the global minimum, and the population will eventually be distributed in the global minimum. It can be seen from Figure 7(b) that the genetic algorithm in MATLAB software improves the BP neural network. The blue curve is the iterative training result of the BP neural network without genetic algorithm optimization. Although after about 100 iterations, the error can tend to converge, the error value is still large. The red curve is the neural network training result optimized by the genetic algorithm. The error is small and only about 60 iterations can converge. It can be seen from the comparison that the genetic algorithm has an obvious optimization effect on the BP neural network.

### 4.2. GA-BP Neural Network Model to Evaluate the Results and Analysis of the Mechanical Properties of Materials

Neural network training requires a large number of training samples, so we randomly select 120 groups of 196 sets of AZ31 and AZ91 magnesium alloy data obtained from the experiment as training samples and confirmation samples and normalize the data for network training. Using the established three-layer BP neural network model to simulate the UTS of AZ31 and AZ91 magnesium alloys, the training results of the comparison sample and the output sample are shown in Figure 8(a). The average error with the comparison value reached 7.3%, and the effect is not ideal. The reason is that the data of different magnesium alloys are highly discrete, which leads to large errors in the conclusion. The data and neural network model should be further adjusted. For the training sample data, a genetic algorithm is used to perform coding selection crossover and mutation processing, to obtain a relatively high target fitness value population. Based on the optimized weight domain value data and parameters, AZ31 and AZ91 magnesium alloys are reestablished with extrusion temperature, extrusion rate, extrusion ratio, solution temperature, and solution time as input. UTS is the output based on the 5-8-1 three-layer BP neural network forecast model optimized by the genetic algorithm, and we select 120 sets of sample data for training. The experimental samples and output samples of the BP neural network optimized by the genetic algorithm are shown in Figure 8(a).

RETRACTED

The UTS differences caused by different stretching times under the same conditions are used to quantitatively characterize the level of tensile performance in the mechanical properties and finally the network is verified by predicting samples. After the BP neural network forecast model optimized by the genetic algorithm is trained, the absolute average error of UTS is reduced from 12.3% to 4.3%, and the maximum absolute error is less than 3%. The error curve of UTS is shown in Figure 8(b).

It can be seen from the figure that, compared with the traditional BP neural network prediction model, the error value fluctuation of the optimized neural network is significantly smaller, and it has higher prediction accuracy. The reason is that the BP neural network optimized by the genetic algorithm significantly increases the fitness value of the sample value and reduces the dispersion of the sample data. The overall optimization avoids falling into the local extreme value and reaches the predetermined value in a short time. The error is small with the experimental value.

From the above analysis, it can be seen that the genetic algorithm is used to optimize the BP neural network model, which further reduces the average error of the model prediction so that the model has more accurate prediction capabilities. The genetic algorithm optimizes the fitting of the true value of the neural network and the predicted value. The curve is shown in Figure 9.

RETRACTED

Compared with the traditional BP neural network data regression, the BP neural network sample data optimized by the genetic algorithm has less discreteness, higher fitness value, and more accurate prediction results. The average error of UTS of AZ31 magnesium alloy is reduced to 0.88%; the average error of YS of AZ31 magnesium alloy is reduced to 3.3%; and the most obvious is that reducing the elongation of AZ31 ELO, the error was reduced to 8.1%, which played a very good optimization effect. Compared with the general BP neural network prediction model, it has higher prediction accuracy.

## 5. Conclusion

In order to predict and evaluate the mechanical properties of magnesium alloy materials, based on the analysis of the structure and mechanical properties of magnesium alloy materials, the 5-8-1 BP neural network prediction model is selected to predict the mechanical properties of AZ31 and AZ91 magnesium alloys. By collecting and sorting out 196 sets of mechanical property data samples in the experiment, it is established that AZ31 and AZ91 magnesium alloys take the extrusion temperature, extrusion rate, extrusion coefficient, solution temperature, and solution time as input. The 5-8-1 three-layer BP neural network prediction model optimized based on the genetic algorithm with UTS, YS, and ELO as outputs. The default value provided by the MATLAB platform changes with the number of iterations so that the BP neural network optimized by the genetic algorithm has a reasonable training time and number of training times. The relative error of the output value and the expected value is relative to the traditional BP neural network optimization. Compared with the error, the prediction effect has been significantly improved, which is basically consistent with the experimental results.

## Figures and Tables

**Figure 1:** The overall structure of the magnesium alloy material mechanical performance evaluation algorithm.

**Figure 2:** BP neural network structure.

**Figure 3:** Schematic diagram of genetic algorithm solving problem. (a) GA search algorithm. (b) Population evolution. (c) Changes in population fitness during evolution.

**Figure 4:** A bit of crossover and mutation genetic example diagram. (a) Cross inheritance. (b) Examples of variance inheritance.

**Figure 5:** Structure diagram of BP neural network model for the evaluation of mechanical properties of magnesium alloy materials.

**Figure 6:** Genetic algorithm to optimize BP neural network flowchart.

RETRACTED

**Figure 7:** Iterative training structure and path of BP neural network and GA-BP neural network. (a) Minima areas of BP network. (b) The error comparison between BP and GA-BP.

**Figure 8:** BP and GA-BP prediction value and its error comparison. (a) The prediction results comparison and (b) prediction comparison between BP and GA-BP.

**Figure 9:** The fitting curve of the true value and predicted value of GA-BP neural network. (a) UTS. (b) YS. (c) ELO.

**Table 1:** Statistical table of processing parameters in magnesium alloy material data samples.

Serial number	Process parameters	Maximum	Minimum	Sample mean
1	Extrusion temperature	418°C	210°C	370°C
2	Squeeze coefficient	78	8	43
3	Extrusion rate	7.8 m/min	0.8 m/min	4.3 m/min
4	Solution temperature	710°C	0°C	420°C
5	Solution time	39 h	0 h	18 h

## Data Availability

The data used to support the findings of this study are available from the corresponding author upon request.
